The article "Potential of Soft-Shelled Rugby Headgear to Reduce Linear Impact Accelerations" was published in 2021. Journal: J Healthc Eng.

# Potential of Soft-Shelled Rugby Headgear to Reduce Linear Impact Accelerations

**DOI:** 10.1155/2021/5567625

**Published:** 2021-04-23

**Authors:** Nick Draper, Natalia Kabaliuk, Danyon Stitt, Keith Alexander

**Affiliations:** ^1^School of Health Sciences, University of Canterbury, Christchurch, New Zealand; ^2^Department of Mechanical Engineering, University of Canterbury, Christchurch, New Zealand

## Abstract

The purpose of this study was to examine the potential of soft-shelled rugby headgear to reduce linear impact accelerations. A hybrid III head form instrumented with a 3-axis accelerometer was used to assess headgear performance on a drop test rig. Six headgear units were examined in this study: Canterbury Clothing Company (CCC) Ventilator, Kukri, 2^nd^ Skull, N-Pro, and two Gamebreaker headgear units of different sizes (headgears 1–6, respectively). Drop heights were 238, 300, 610, and 912 mm with 5 orientations at each height (forehead, front boss, rear, rear boss, and side). Impact severity was quantified using peak linear acceleration (PLA) and head injury criterion (HIC). All headgear was tested in comparison to a no headgear condition (for all heights). Compared to the no headgear condition, all headgear significantly reduced PLA and HIC at 238 mm (16.2–45.3% PLA and 29.2–62.7% HIC reduction; *P* < 0.0005, *η*_p_^2^ = 0.987–0.991). Headgear impact attenuation lowered significantly as the drop height increased (32.4–5.6% PLA and 50.9–11.7% HIC reduction at 912 mm). There were no significant differences in PLA or HIC reduction between headgear units 1–3. Post hoc testing indicated that headgear units 4–6 significantly outperformed headgear units 1–3 and additionally headgear units 5 and 6 significantly outperformed headgear 4 (*P* < 0.05). The lowest reduction PLA and HIC was for impacts rear orientation for headgear units 1–4 (3.3 ± 3.6%–11 ± 5.8%). In contrast, headgear units 5 and 6 significantly outperformed all other headgear in this orientation (*P* < 0.0005, *η*_p_^2^ = 0.982–0.990). Side impacts showed the greatest reduction in PLA and HIC for all headgear. All headgear units tested demonstrated some degree of reduction in PLA and HIC from a linear impact; however, units 4–6 performed significantly better than headgear units 1–3.

## 1. Introduction

Rugby Union is a popular contact sport played by approximately 8.5 million people in over 121 countries worldwide [1]. The collisions inherent in the game can impart large forces and accelerations to the head during contact. Studies conducted into the forces experienced by the head during gameplay found average peak linear accelerations (PLA, measured in g force) to be in the region of 10–38 g [2–7], with some reaching PLA values of up to 103–165 g [2–5, 7, 8], and a consistent number greater than 80 g [5]. Given rugby's high reported impact accelerations, players are at a much higher risk of injury compared to noncontact sports [9]. One of the most common injuries in rugby is concussion [10–13] with incidence rates ranging 0.4–46/1000 match hours [14–20]. These incident rates are typical across all levels (amateur, college, subelite, and elite) for both women's and men's rugby [16–21]. Furthermore, concussion-related injuries account for 25% of all days lost from rugby participation [13].

Increased attention on the negative effects of sports concussions and recent advances in technology have resulted in a number of innovative theoretical approaches being developed in order to analyse impacts in a sports context [22, 23]. Approaches have to include laboratory simulations, human tests, and tests with animals [22–25]. Whyte et al. (2019) provided a comprehensive review of impact testing for sports headgear and highlighted the need for experimental validation in all theoretical approaches [23]. In accordance with these research innovations, our research approach is focussed on the potential of soft-shell headgear to reduce peak linear accelerations [24, 25].

Peak linear acceleration represents a commonly reported measure of impact intensity. Alternatively, the head injury criterion (HIC) has been increasingly used to estimate the likelihood and severity of brain trauma. The HIC has gained popularity because it focuses on the severity index on the part of the impact most likely to be relevant to the risk of injury to the brain [26]. This is achieved by averaging the integration of the resultant acceleration versus time curve over whatever time interval yielding the maximum value of HIC. In 1998, the National Highway Traffic Safety Administration introduced HIC_15_, where *t*_2_ and *t*_1_ are no more than 15 ms apart [27]. There are currently, however, no accepted HIC thresholds for mTBI or concussion likelihood. Despite this, the HIC score provides a useful method through which different impacts and their severity can be assessed [73].

When the head experiences impact accelerations, differences in density cause parts of the brain to accelerate at different rates, causing stresses and strains within the brain tissue [28]. This can lead to neuronal and axonal damage [28]. The brain can handle some deformation; however, once a certain threshold is surpassed, trauma occurs which can elicit a variety of biological responses [28]. These may be structural (torn vessels and axons) or functional (changes in blood flow or neurological status) and may be immediate or delayed [28]. This gives rise to the short-term symptoms of concussion such as loss of balance and memory [28]^.^ Concussions and other head injuries can result in changes to the integrity of gray and white matter [28].

The developing brain is more susceptible to concussion than the adult brain and may require more time to recover [29]. Impacts over 10 g that do not result in a participant presenting with acute symptoms of concussion have been classified as subconcussive impacts [30]. Repetitive subconcussive impacts have been implicated as an additional long-term health risk [31]. It has been suggested that concussions, or combinations of concussions and subconcussive head impacts, may result in long-term conditions such as chronic traumatic encephalopathy [32], mild cognitive impairment [33], and depression [34]; however, the exact mechanisms resulting in these conditions are yet to be fully elucidated.

Despite the potential health implications, concussions often go unreported [35, 36]. In some instances, concussions can go unreported until symptoms start to show, which can be several days later [35]. Concussive head impacts often do not result in a loss of consciousness, which can further complicate the diagnosis of a concussive injury on the field [35]. It has been reported that approximately 90% of concussions do not result in a loss of consciousness [36]. As a consequence, concussion underreporting rates are estimated to be as high as 50%–90% [36]. These generate an estimated economic burden of $60 billion annually in the US alone [37].

Given the health risks associated with concussive and indeed subconcussive impacts, developments within the game that might mitigate these risks would be important for the future of the game. One source of risk mitigation might be realised through the use of soft-shell headgear. Until recently, World Rugby (WR) permitted one class of headgear, with specifications imposed on thickness (10 + 2 mm max) and density (60 kg/m^3^ maximum density; 45 + 15/m^3^ tolerance band) [38]. All rugby headgear had to meet these specifications and receive approval in order to be suitable for the gameplay [38]. In 2019, World Rugby introduced a medical device trial process allowing headgear to meet more flexible criteria and to be considered for use in gameplay, irrespective of the previous regulations [39].

At present, N-Pro headgear is the only headgear to gain WR approval through this new process. Despite the mounting literature suggesting that headgear can reduce impact accelerations and potentially concussion risks [24, 40–42], the use of rugby headgear remains optional, with few players actively wearing them. Reasons cited for not being used by players include views that they offer little increase in safety, interfere with gameplay, and are not worth the money [43].

Rugby Union is New Zealand's national game, the second most popular sport for young people [44], and is quickly gaining popularity worldwide [1]. As a consequence, protecting players from the long-term effects of concussion is perhaps imperative for the future of the sport. Until recently, manufacturers stated that rugby headgear was designed only to protect against cuts and scrapes. The change in the laws by WR means that there are new types of headgear coming onto the market which claim impact acceleration reduction (N-Pro, Gamebreaker) [24, 45, 46] and which, therefore, have the potential for concussion mitigation. The need for clear data on whether or not headgear can make a difference in reducing head accelerations and associated injury risks is more important now than ever. Therefore, the aim of this study was to examine the effectiveness of three popular soft-shelled rugby headgear units and two of the newer headgear units in reducing peak linear accelerations and the HIC score.

## 2. Materials and Methods

### 2.1. Headgear Units

Five models of headgear (and a total of 6 headgear units) were chosen: CCC Ventilator, Kukri, 2^nd^ Skull, N-Pro, and a medium and large-sized Gamebreaker Pro (Figure 1) (herein referred to as headgears 1–6, respectively) with all units in medium size except headgear 6. Headgear units 1 and 3 comprised light weight (≤45 kg/m^3^) polyethylene foam arranged in cells around the headgear to provide padding. For headgear unit 1, the foam was formed from honeycomb shaped cells whilst in headgear 3 the cells were ʊ shaped. Headgear unit 2 was formed from a light weight (≤45 kg/m^3^) ethylene vinyl acetate (EVA) foam arranged in cells similar to headgear 1. Headgear 4 was manufactured using a thicker, higher density (≥45 kg/m^3^) open-cell polyurethane foam arranged in square cells of varied size [44]. Headgear units 5 and 6 were composed of EVA foam and a layer of impact-absorbing foam developed by D3O® (≥45 kg/m^3^) [47]. Headgear units 1–3 were manufactured from closed-cell foams, whilst units 4–6 comprised foams that are viscoelastic and open celled. Headgear units 5 and 6 were the thickest samples (15–20 mm max thickness), when compared with headgear unit 4 (12–13 mm max thickness) and headgear units 1–3 (8–10 mm max thickness).

All headgear units had a tight fit on the head form with no slippage to ensure a consistent impact region throughout testing. All headgears were new and in unused condition. Headgear units 1–4 had been World Rugby approved and allowed to be used during gameplay; however, headgear units 5 and 6 are still undergoing assessment by WR. It should be noted that World Rugby-approved headgear (prior to the law 4 trial approval process) was not designed to mitigate risks of brain injury or skull fracture.

### 2.2. Testing Protocol

The testing of the headgear units was carried out using a twin wire-guided, gravity-induced drop test rig. A 50^th^ percentile male head form (Humanetics Innovative Solutions Inc.) was used to simulate a player's head, on which the headgear was mounted (Figures 1 and 2). The head form was instrumented with a three-axis accelerometer (MEAS 53–0500, ±500 g, 10 kHz sampling rate) held at the centre of gravity of the head form. The head form and sensors were calibrated using the protocol set by the code of Federal Regulations (CFR) [48]. A 1 inch (25 mm) Modular Elastomer Programmer (MEP) pad by Cadex Inc. served as an impact surface (Figure 2). The pad was calibrated at an independent laboratory by Cadex Inc. Impact locations were determined using the NOCSAE [45] and World Rugby standards [34] for impact testing of sporting headgear (Figure 2). The top of the head (crown) was excluded from testing as preliminary impacts showed similar PLA and HIC reduction to other areas. Additionally, of the impact locations described in the standard, the crown is the least commonly impacted area during gameplay [5, 7, 49]. The head form was dropped from 4 different heights, corresponding to 13.8 J impact energy, specified by World Rugby [38], 300 mm drop height specified by World Rugby and common in previous studies [24, 38, 39, 41], and heights providing impact velocities of 3.46 and 4.23 m/s specified by NOCSAE [45]. These drop heights are summarised in Table 1. Impact velocities were verified to ±2.8% of calculated values using high-speed imagery prior to testing.

The impact energy was determined for the total falling mass of 5.9 kg including the drop frame (Figure 2). Five repeats for each orientation and drop height were performed with 60 seconds between successive drops [50].

It should be noted that this study did not intend to exactly replicate either the World Rugby or NOCSAE standards but used them as a guideline from which to extend the investigation of headgear behaviour. This study did not test headgear for World Rugby approval but assessed and compared the impact attenuation behaviours of selected headgear. Prior to testing the headgear units, a no headgear baseline trial was completed with PLA and HIC measurements assessed and calculated at each drop height. In the analysis of the headgear units, comparisons were made between PLA and HIC results in the no headgear condition and PLA and HIC scores for each of the 6 headgear units.

### 2.3. Data and Statistical Analysis

Linear impact accelerations were measured for each drop. These were recorded 5 ms before a 10 g threshold was reached and continued recording for 50 ms thereafter. Initial trials found this to encapsulate the entire acceleration-time curve for the longest impact times recorded. Data was then processed in a custom MATLAB code to identify the peak acceleration and maximum HIC value for each of the five repeats. HIC_15_ was calculated using the following equation:

(1) $$\begin{array}{c} \text{HIC}=\left(t_{2}-t_{1}\right){\left[\frac{1}{t_{2}-t_{1}}\int_{t_{1}}^{t_{2}}a\left(t\right)dt\right]}^{2.5},\left(\begin{array}{ccc} a_{11} & \ldots & a_{1n}\\ \vdots & \ddots & \vdots \\ a_{m1} & \cdots & a_{mn} \end{array}\right) \end{array}$$

where *t*_2_ – *t*_1_ = 15 ms. Mean PLA and HIC values were calculated for each headgear unit at each drop height in each orientation. Composite averages were taken as the average PLA and HIC across all orientations for each headgear across three heights (238, 610, and 912 mm). Distributions, descriptive statistics, and mixed-design ANalyses Of VAriance (ANOVA) were calculated using SPSS (Version 25, IBM SPSS Statistics Inc., Chicago, IL, USA). Data were assessed for violations of the assumptions of normality of distribution using the Shapiro-Wilk test, with results showing Gaussian distribution. An alpha level of *P* < 0.05 was set for accepting statistical significance. Cohen *d* and partial eta squared (*ɳ*_p_^2^) were used to assess size effect where the values of 0.2, 0.5, and >0.8 represent small, moderate, and large differences and 0.05, 0.10, and >0.20 represent small, intermediate, and large effect, respectively. The drop height of 300 mm was excluded from the composite statistical analysis, as 238 mm and 300 mm impact behaviours follow the same trend and displayed similar PLA and HIC values. The 300 mm drop height was, however, included in location-specific analyses of the data.

## 3. Results

### 3.1. Composite Behaviour

Descriptive data for PLA and HIC along with percentage reductions in PLA and HIC can be found in Tables 2 and 3, respectively. Results of a mixed-design ANOVA indicated that all headgear significantly reduced the PLA values when compared with the no headgear condition at all heights (*P* < 0.0005, *η*_p_^2^ = 0.987–0.989). There were no significant differences in PLA between headgears 1–3 at any of the three heights. Post hoc testing results indicated that headgear unit 4 significantly reduced PLA when compared to headgears 1–3 at all three drop heights. Furthermore, headgear units 5 and 6 reduced PLA significantly more than headgear units 1–4 across all heights (*P* < 0.05). Headgear unit 6 produced a significantly greater PLA reduction when compared to headgear unit 5 at 238 mm drop height (*P* < 0.05). At all heights above this, neither unit 5 nor 6 significantly reduced PLA more than the other; however, they consistently outperformed reductions in PLA seen for headgear units 1–4.

Following a similar trend to PLA, results from a mixed-design ANOVA indicated that all headgear units significantly reduced HIC when compared to the no headgear condition at all heights (*P* < 0.0005, *η*_p_^2^ = 0.988–0.991). Post hoc testing indicated that at the 238 mm drop height, headgear unit 1 reduced HIC significantly more than headgears 2 and 3 (*P* < 0.05). No significant difference in HIC reduction between headgears 1–3 was seen at any other height (Table 3). Following the trend of PLA reduction, headgear unit 4 significantly reduced HIC when compared with headgear units 1–3, and both headgear units 5 and 6 significantly reduced HIC compared to all other headgear units 1–4 (*P* < 0.05). At 238 mm, headgear 6 reduced HIC significantly more than headgear 5 (*P* < 0.05). This was not observed at any other heights.

### 3.2. Location-Specific Behaviour

As can be seen in Figures 3 and 4, all headgear reduced average PLA and HIC to some extent. The average PLA (Figure 3) and HIC values (Figure 4) were the highest for rear impacts across all headgear at all heights. Side impact locations showed higher average PLA and HIC scores than the forehead, front boss, and rear boss locations. Forehead and rear boss impact locations showed similar average PLA and HIC values across all heights whilst both gave consistently lower values than side and rear impacts. Front boss impacts gave the lowest PLA and HIC across all heights and headgear units. The same trend was observed in the no headgear condition. Headgear 4 showed higher mean PLA and HIC values than headgear units 5 and 6 in rear impacts, but lower than headgear units 1–3.

Table 4 shows the average percentage of PLA and HIC reduction across all four drop heights for each orientation. For headgear units 1, 3, and 4, the least PLA and HIC reduction occurred in the rear orientation, whilst the remaining headgear displayed the least PLA and HIC reduction in the front boss orientation. It should be noted that the difference in PLA and HIC reduction between the rear and front boss impact locations is minimal for all headgear with the exception of headgear unit 4. All headgear displayed the highest PLA and HIC reductions in side, forehead, and then rear boss orientations. Headgear units 4–6 consistently display larger PLA and HIC reductions across all positions compared to headgear units 1–3.

## 4. Discussion

The aim of this study was to examine the potential of soft-shelled rugby headgear units to mitigate peak linear accelerations and HIC scores. All headgear units reduced PLA and HIC scores when compared to the no headgear condition. This was perhaps to be expected as the presence of foam padding extended the time of total deceleration, thereby decreasing the peak acceleration. Headgear performance was clearly split into two groups: headgear units 1–3 and units 4–6. Headgear units 1–3 were composed of lightweight (≤45 kg/m^3^) closed-cell foam [41, 51], which measured between 8 and 10 mm max thickness, to provide impact attenuation. All three incorporated very similar materials, at similar thicknesses, in similar cell structure arrangements across the headgear. This is likely why all three display similar impact attenuation behaviour. In contrast, headgear unit 4 was manufactured using a high density, viscoelastic, open-cell polyurethane foam [24] whilst headgear units 5 and 6 were composed of a layer of EVA foam [45] and a layer of impact-absorbing, viscoelastic foam developed by D3O® [45]. Headgear units 4–6 each have a higher total thickness than headgears 1–3. Headgear units 4–6 lowered PLA and HIC significantly more than headgears 1–3 across all impacts; however, headgear units 5 and 6 lowered PLA and HIC significantly more than headgear unit 4 across all impacts (*P* < 0.05). The difference between headgear unit 4, when compared with units 5 and 6, can likely be attributed to the difference in thickness, given that headgear units 5 and 6 were thicker than headgear unit 4.

Side impacts showed the highest PLA and HIC reduction for all headgear units as the side of the headgear had the largest single surface area of foam involved in the impact when compared to all the orientations tested. Headgear units 1–4 showed their lowest impact attenuation in the rear orientation. These headgear units have laces at the back to ensure a tight fit when worn. As a consequence, there is less padding in that area. Headgear 4 has a higher thickness of material than the other lace-up types, and therefore, this unit reduced PLA and HIC slightly more than headgear units 1–3 in the rear orientation. Headgears 5 and 6 use a large elastic tube with a foam insert instead of laces, thereby providing higher impact attenuation than the other headgear units in the rear orientation. Front and rear boss impact positions performed better than rear impacts, but not as well as the side or forehead due to having lower amounts of foam involved in the impact compared to side and forehead, but more than the rear.

Studies of impact locations during gameplay all report the side of the head as the most commonly impacted region, followed by the front and back (with similar impact frequencies), and lastly the top of the head (crown) [5, 7, 49]. It is unknown if the higher impact attenuation behaviour of the side impact location is intentionally designed into the headgear from results of previous field investigations or simply a consequence of the curvature of the head allowing for a flatter impact surface (therefore larger foam area involved in impact). Despite the back of the head being a common location for collision impacts, most of the headgear units in our study had gaps in padding at the back of the head. Impacts directly to the back of the head must be a concern for players, coaches, and health professionals given that it is a common collision point in gameplay. Headgear units 5 and 6 had an increased depth of foam in this orientation, thereby offering the greatest degree of PLA and HIC mitigation when compared with units 1–4 [5, 7, 49].

Headgear unit 6 (large) consistently performed better than headgear 5 (medium). The medium size fit very tightly on the head form and consequently some degree of precrushing of the foam would have been present on the medium headgear, thereby reducing the amount of deformation the foam could undergo during impact. Additionally, the larger-sized headgear would have had, albeit minimally, a greater area of foam involved in the impact, therefore increasing the amount of energy absorbed in each impact. These differences were consistent, but nonsignificant at heights above 238 mm.

All headgear units demonstrated a lowering of attenuation effectiveness with increasing drop height. The foams contained within each of the headgear units can only absorb a certain amount of energy through deformation. This amount of energy depends on a range of structural properties intrinsic to the material involved as well as the thickness of the material. As impact energy increases, the foam dissipates a lower percentage of the total energy involved; it is less effective at high impact energies. The higher density, viscoelastic, open-cell foams used in headgear units 4–6 were observed to dissipate a much greater proportion of the impact energy than the lower density closed-cell foams used in units 1–3. Closed-cell foams are comprised of many tiny pockets of air trapped within cells made of the foam polymer. Energy is absorbed through compression of the air pockets inside and deformation of the cell walls giving the foams their ‘springy' feel when compressed. In open-cell foams, cells are not fully closed off, allowing air to move through the material. In these, energy is absorbed through the deformation of the polymer structure. As this happens, the air is pushed through the cellular structure, offering some resistance to deformation. Open-cell foams are less stiff than the equivalent density closed-cell foams; therefore, much higher density foams can be used in ‘soft-shelled' headgear than would be possible with closed-cell foams. This increased foam density, as well as increased viscoelastic nature of the open-cell foams, likely accounts for much of the difference in impact attenuation exhibited by the two foam types.

The headgear using closed-cell foam experienced significant degradation in areas when subjected to the highest energy impacts. This was likely due to a bursting of the cell walls encapsulating the air pockets. This degradation was limited to headgear units 1–3 but only occurred in the forehead and front boss areas, where there was a lower area of foam involved in the impacts. This was not observed in the other headgear units.

Our data suggest that soft-shell headgear has the potential to reduce the risk of concussive head injuries. If the accelerations seen in an impact can be lowered, the concussive injury risk could potentially be reduced. The mechanisms of concussion, specifically the causation pathway and the effect of an impact on the underlying mechanisms in the brain, are yet not fully understood; however, the link between high-intensity head impacts and concussion is recognised [10, 13, 20, 31]. The results of our study suggest that the headgear tested could potentially lower linear impact accelerations by up to 50% which could provide a degree of protection for players. Further testing of headgear performance on the field would be required before any definite conclusions could be drawn on their protective performance. Additionally, the effect of the fit of the headgear would need to be investigated with regard to the impact attenuation behaviour.

Importantly, our study was limited to linear accelerations and the degree of mitigation realised by soft-shell headgear in a laboratory setting. Further investigation is needed investigating rotational accelerations and their role in concussive injuries. Recent research indicates that rotational accelerations may be more damaging to the brain than linear and may be more prevalent in rugby collisions [28, 52]. At present, however, no accepted method exists to quantify the rotational accelerations. A method similar to HIC has been proposed which integrates the rotational and linear acceleration [10, 52]; however, validation standards do not yet exist for this method. Further investigation is needed regarding the metrics quantifying injury risk using both rotational and linear accelerations and then to examine the potential of current and future soft-shell headgear designs to mitigate both linear and rotational accelerations in collisions in a laboratory setting and in field studies.

## 5. Conclusion

This study provides further evidence regarding 5 commercially available headgear units and their potential to reduce peak linear accelerations and HIC score during the collisions inherent in Rugby Union. The research has application to other codes where such contacts affecting the head are possible, but where a hard shell headgear unit is not permissible within the rules of the game, examples include rugby league and Australian rules football. In our study, all headgear units significantly reduced the PLA and HIC during an impact. The newer designs of headgear (headgear units 4–6) reduced PLA and HIC significantly more than older World Rugby approved headgear (units 1–3). All except headgears 5 and 6 showed little reduction in PLA and HIC in a rear impact, and all headgears showed a reduction in effectiveness at higher drop heights. Further investigation is required into rotational accelerations and their importance in collisions in rugby. In addition, it will be important to establish standards for rotational acceleration assessment and examining the extent that current and new soft-shell headgear models can mitigate both linear and rotational impact accelerations.

## Figures and Tables

**Figure 1:** Headgear involved in the testing from top left to bottom right: headgear 1, headgear 2, headgear 3, headgear 5, headgear 6, and headgear 4.

**Figure 2:** Drop test setup showing the different impact orientations tested (Rear boss, Rear, Side, Forehead, and Front boss).

**Figure 3:** Mean (SD) peak linear acceleration for each headgear unit in each orientation at (a) 238 mm, (b) 300 mm, (c) 610 mm, and (d) 912 mm.

**Figure 4:** Max HIC scores for all headgear units in each orientation from drop heights of (a) 238 mm, (b) 300 mm, (c) 610 mm, and (d) 912 mm.

**Table 1:** Details of the drop heights used.

Drop height (mm)	Impact velocity (m/s)	Impact energy (J)	Authority
238	2.16	13.76	World Rugby
300	2.43	17.24	World Rugby
610	3.46	35.32	NOCSAE
912	4.23	52.78	NOCSAE

**Table 2:** Mean (SD) values for the composite behaviour of the headgear compared to no headgear.

	Peak acceleration (g's)			HIC score		
	238 mm	610 mm	912 mm	238 mm	610 mm	912 mm
No headgear	71 (0.2)	142.6 (2.0)	198.1 (0.8)	100.8 (0.6)	424.5 (4.3)	853.1 (8.3)
Headgear 1	58.2 (1.4)	132.8 (1.6)	184.4 (0.9)	67.8 (2.9)	372.8 (5.8)	743.7 (9.4)
Headgear 2	58.8 (1.0)	131.4 (1.4)	183.2 (2.0)	70.9 (1.6)	363.3 (3.5)	741.9 (13.6)
Headgear 3	60.0 (1.9)	132.1 (2.5)	186.5 (2.8)	71.6 (4.0)	371.7 (11.1)	751.5 (15.2)
Headgear 4	48.3(1.8)	111.7(3.7)	158.6 (6.1)	50.4(3.2)	280.3 (11.4)	572.8 (32.4)
Headgear 5	42.9(1.7)	96.2 (3.8)	136.8 (4.3)	42.9 (2.7)	209.7 (13.7)	435.8 (26.3)
Headgear 6	39.0 (1.7)	93.8 (3.3)	132.4 (4.2)	37.4 (2.3)	201.8 (11.3)	412.1 (19.3)

**Table 3:** Mean (SD) composite percentage reduction values compared to no headgear.

	PLA Reduction			HIC Reduction		
	238 mm	610 mm	912 mm	238 mm	610 mm	912 mm
Headgear 1	18.5 (2.2)	7.2 (2.2)	6.5 (1.2)	32.4 (3.7)	13.3 (2.4)	12.4 (2.2)
Headgear 2	17.8 (1.9)	7.9 (2.2)	7.2 (1.5)	29.7 (3.3)	14.7 (2.4)	12.5 (2.8)
Headgear 3	16.2 (3.0)	7.8 (2.9)	5.6 (1.8)	29.2 (4.8)	14.9 (3.5)	11.7 (2.4)
Headgear 4	32.6 (2.7)	21.5 (3.4)	19.9 (3.1)	50.0 (4.0)	34.7 (3.9)	33.9 (4.6)
Headgear 5	39.7 (3.1)	31.7 (3.5)	29.9 (2.7)	57.3 (4.0)	49.6 (4.5)	47.4 (3.8)
Headgear 6	45.3 (2.6)	33.6 (3.3)	32.4 (2.4)	62.7 (3.1)	51.6 (3.9)	50.9 (2.9)

**Table 4:** Mean (SD) percentage reduction values averaged across all four drop heights for each orientation.

Headgear	PLA					HIC				
	Side	Forehead	F. boss	Rear	R. boss	Side	Forehead	F. boss	Rear	R. boss
1	18.2 (5.4)	12.9 (5.6)	7.8 (3.5)	5.7 (4.7)	11.1 (3.8)	29.3 (9.9)	24.6 (8.0)	14.7 (6.2)	11.0 (8.5)	22.1 (5.1)
2	18.6 (6.3)	14.6 (5.6)	6.3 (3.0)	7.0 (3.1)	10.9 (4.1)	29.1 (10.6)	25.2 (8.1)	11.3 (5.4)	13.4 (4.6)	19.1 (6.4)
3	18 (4.1)	12.7 (4.7)	7.0 (3.4)	3.3 (3.6)	9.3 (2.7)	29.0 (7.5)	25.2 (6.1)	13.6 (6.0)	8.0 (6.9)	18.9 (3.8)
4	36.9 (2.6)	27.7 (7.4)	20.2 (4.0)	11.0 (5.8)	25.2 (3.4)	57.9 (3.6)	44.0 (8.2)	32.5 (3.6)	19.5 (10.6)	41.1 (3.8)
5	49.2 (2.7)	37.1 (7.2)	27.4 (5.7)	33.2 (4.1)	30.6 (3.8)	67.2 (0.7)	57.3 (6.9)	44.7 (6.8)	49.7 (4.9)	46.9 (4.0)
6	50.4 (2.5)	40.8 (7.0)	31.4 (6.4)	34.2 (6.3)	35.2 (4.9)	67.5 (1.6)	60.9 (5.6)	49.2 (7.3)	52.0 (6.8)	51.5 (4.2)

## Data Availability

Access to the data from this study is restricted due to commercial confidentiality.
